The article "Microbiological characterization and effect of resin composites in cervical lesions" was published in 2017. Journal: J Clin Exp Dent.

# Microbiological characterization and effect of resin composites in cervical lesions

**DOI:** 10.4317/jced.52978

**Published:** 2017-01-01

**Authors:** Bonfanti Carlo, Nicola Barabanti, Giorgio Piccinelli, Vicente Faus-Matoses, Antonio Cerutti

**Affiliations:** 1 Institute of Microbiology, Department of Molecular and Translational Medicine, University of Brescia, Brescia, Italy; 2 Tutor, Department of Restorative Dentistry, University of Brescia, Italy; 3 Institute of Microbiology, Department of Molecular and Translational Medicine, University of Brescia, Brescia, Italy; 4 DDS, MSc. Master of Restorative Dentristy and Endodontics, Department of Stomatology, Medicine and Dental School, Valencia University, Spain; 5 Professor, Department of Restorative Dentistry, University of Brescia, Italy

## Abstract

**Background:**

Non carious cervical lesions associated to muscle hyperfunctions are increasing. Microhybrid resin composites are used to restore cervical abfractions. The purpose of this study was to investigate if resin composites modify tooth plaque, inducing an increment of cariogenic microflora and evaluate their effect, *in vivo* and *in vitro*, against *S. mutans*.

**Material and Methods:**

Eight abfractions were restored with two microhybrid resin composites (Venus, Heraeus-Kulzer® and Esthet-X, Dentsply®), after gnatological therapy, in three patients with muscle hyperfunctions. For each abfraction three samples of plaque were taken from the cervical perimeter: before the restoration, one week and three months after restoration. The samples were evaluated both by traditional microbiological methods and by Polymerase Chain Reaction (PCR). *In vitro*, disk-shaped specimens of the two composites were prepared to estimate the effects against pre-cultured *S. mutans*, after incubation at 37°C for 24h and assessed by a turbidimetric technique.

**Results:**

*In vivo* no differences were found in plaque growth, for all samples, before and after restoration with both composites; *in vitro*, instead, a significant reduction of *S. mutans* growth was found between specimens of two composites (Mann-Whitney U-test *p*>0,06).

**Conclusions:**

In this study a relevant consideration was elicited: composite materials, *in vivo*, do not modify plaque composition of non carious cervical lesions to a potential cariogenic plaque.

** Key words:**Abfraction, restoration, S. mutans, composite, class V.

## Introduction

Non carious cervical lesions are a well known problem for every dentist, but which is not always simple to be solved.

There are different kinds of cervical lesions: erosions, brushing lesions, mechanical lesions and abfractions.

Abfractions were first studied by Grippo (1,2), their aetiology have been unknown for over twenty years. Rees (3) and his colleagues, the best experts of this kind of lesion, have found a relation between abfraction and occlusal charge.

Cervical lesions are characterized by a loss of mineralized dental tissue, in the zone of cement-enamel junction, with no carious process.

Abrasions are due to mechanical forces and they consist of a loss of cervical dental tissue, because of repeated and wrong friction of objects or materials on the surface of the teeth. Food, toothbrush bristles, abrasive toothpaste, wrong toothbrushing, incorrect use of dental floss are some of the causes of abrasions. The first tissue attacked by abrasions is cement, because it is 29 times less resistant than dry enamel. During time we witness a loss in both inorganic and organic components, associated to remineralization and dentinal sclerosis process.

The general aspect of this kind of lesions is a polish concave lesion located on the buccal surface of a few adjacent teeth; they appear smooth, with clean-cut margins and with a variable depth depending directly on the length and the intensity of the traumatic ravage. The over thirty age group is the most struck. Such lesions are more frequent in the arch opposite to the habitual hand used during personal hygiene, mostly on premolar and molar teeth.

Erosions consist of a progressive dissolution of dental structure, cervical and not, due to non bacterial exogenous/endogenous chemical agents. Among exogenous factors there are soft drinks; in particular, juices and fizzy drinks are the most involved in erosion. Such drinks are rich in phosphoric acid and overall of citric acid that are able to chelate, and consequently to dissolve, calcium ions of dental tissues. Low alcoholic strength spirits (such as wine, fizzy, beer, etc) have an intrinsic erosive power and, if assumed in excessive amount, they cause vomiting, which contributes to the acidification of the oral cavity.

The abuse of some narcotic substances, like amphetamines (ecstasy in particular), determines dehydration and as a consequence, hyposalivation, stimulating the urge to drink huge amounts of liquids in the form of low pH soft drinks.

The main endogenous source of acids is represented by gastric juices (rich in HCl, chloridric acid) which are able to enrich the oral cavity in consequence of gastricoesophageal reflux or spontaneous vomiting or induced voluntarily by bulimics.

Patients affected by food disorders, in particular, anorexia or bulimia, who frequently vomit, show erosive lesions located selectively on palatal surfaces of upper teeth, on occlusal ones and on gingival third areas. On the other hand, buccal cervical lesions that can be found in bulimics and anorexics, are not due to vomit events but to the intake of huge amounts of low pH soft drinks and fresh fruits with the aim of reducing thirst and of inducing diarrhoea.

As observed for decays, mouth dryness, apart from its aetiology, fosters the erosive process, because the acids which reach the oral cavity are poorly watered down and inadequately buffered.

Chronic alcoholism is another frequent cause of erosion by exogenous acids because it is often associated with gastritis and regurgitation.

Clinical cases of erosions are noticed as a loss of dental tissue on numerous teeth, both on palatal-lingual and buccal sides. Acid erosion dissolves huge portions of the tooth; the lesions result in a poor depth with rather detectable margins, without sharp angles; dentinal structure is hard and with a glassy aspect.

Abfractions are non-carious cervical wedge-shaped lesions, due to biomechanical occlusal stresses which exert abnormal forces of compression, torsion and flexion on the tooth, bringing about delaminating of the enamel and loss of cervical tooth tissue. Lesions result in wedge-shaped acute angles with the apex facing the pulp chamber, often subgingival. Dental tissues appear glassy, brown-yellow and of hard consistence because of apposition of secondary (sclerotic) dentine. Grippo (1) was the first clinician who investigated this kind of lesion; he tried to point out their aetiology and proposed to classify abfractions in cervical lesions. Grippo *et al.* (4) have revisited nomenclature, definitions and classification for tooth surface lesions. Rees JS, Hammadeh M (5), Litonjua *et al.* (6), Rees and Jagger DC (7), studied abfraction biomechanical formation by means of finite element analysis and photoelastic models showing stress concentration at the dental cervical area, using different strategies of loading. Even if the main cause of abfraction formation is related to bite forces, the actual pathogenesis remains controversial. Rees (7) suggested for abfraction aethiology an involving of undermining of the cervical enamel along the amelodentinal junction and the different thickness of periodontal ligament and alveolar bone of the teeth. Furthermore they observed abfractions on anterior teeth: incisors, canines and premolars above all in the upper arch. In our observations, instead, we noticed a greater presence of non-carious cervical lesions in premolars both in the lower and in the upper arch; additionally, these lesions were associated with signs of wear on the occlusal surfaces of the teeth in patients who suffered from muscle hyperfunction. The purpose of our study was not to analyse the dynamics of abfraction formation but to investigate the changes in microbiological flora before and after the restoration of cervical lesions. In order to be sure that our microhybrid composite restorations would last over time and would not be overloaded by bite stresses.

We collaborated with Prof. Bodin, professor of Gnathology in our University and together we established a gnathological therapy by means of a bite before starting conservative therapies.

Problems involved in cervical lesion:

Cervical lesions of any nature create aesthetic defects of teeth and even if pulp odontoblasts react producing secondary dentine, sometimes patients complain about hypersensivity due to loss of dental tissues.

Not as often as we might imagine this kind of lesions ends up in decay, in particular abfractions. This is not an impossible event, because decay disease is a multifactorial disease in which the site of the defects on the tooth has an important role.

Another problem extensively studied by the scientific community (8-13) was about which restorative material should be used for solving aesthetic cervical lesions: ionomer-glass, compomers, composite, resin-modified glass-ionomers. In our opinion the most important aim is to analyse all kind of cervical lesions and investigate their aetiology in order to complete a correct diagnosis and to apply the most adequate material. Microhybrid composites are nowadays the most performant materials in dentistry because of their chemical and physical characteristics, but to improve their qualities we have to eliminate first the causes that are involved in cervical lesions and to work with a strict restoration protocol.

## Material and Methods

We have performed both an *in vivo* and an *in vitro* research.

-*In vivo* study

In the *in vivo* study we analysed eight cervical lesions in three patients with abfractions associated to muscle hyperfunctions, in gnatological therapy. In each patient two or three lesions were restored with two different resin composites. Four of these lesions were restored with Venus microhybrid composite (Heraeus-Kulzer®) and four with Esthet-X (Dentsply®). For each lesion two plaque samples were taken before the restoration, two samples were taken after a week and two a month after restoration. Two plaque samples were taken from a sound tooth too as control. A plaque sample was taken by a periodontal probe from the cervical perimeter of the lesion, then put into a test tube and mixed with 0.5ml of physiological solution.

These samples were evaluated by traditional microbiological method in different cultural plates: blood-agar medium, Mitis salivarius medium and Mitis salivarius with bacitracin medium, more selective for *S. mutans*. Six plates for each sample (three plates in aerobiosis and three in anaerobiosis), were incubated for 24h at 37°C. After incubation a sample from each plate was taken and evaluated by optical microscopy on a slide to detect a the presence of *S. mutans* and other bacteria.

Another kind of plaque sample was taken with an ISO 40 paper cone to be evaluated by Polymerase Chain Reaction (PCR) technique. The paper cone was kept for 10 seconds on the lesion perimeter without deepening up to 2 mm in periodontal sulcus. The cones were maintained in test tubes at -20°C up to the end of the sample collection. Then all these samples were processed for PCR, by Symbiosis® technique for the extraction of DNA from the cones: the DNAs were amplified and their products were migrated on agar gel to evaluate, in comparison to *S. mutans* DNA marker, the presence of such bacterium in the cervical lesions or in their restorations.

Restorative execution: after polishing the surface to be restored with a rubber bur on a contra-angle to eliminate the exceeding plaque (patients were asked not to clean their teeth for a 24h time), we chose the fitting tooth colour, using the respective colour scales provided by the two firms: Heraeus-Kulzer® 2Layer scale and Dentsply® TruMatch scale. A rubber dam was applied. We used a round-shaped diamond bur (Komet®) on a high-speed handpiece to polish the cavity and prepare a bevel on the enamel surface. Such bevel consisted of a 30°-45° in angulations, 3 mm in length: cervical enamel, where possible, was maintained. We etched with 37% phosphoric acid for 30 seconds on enamel and for 15 seconds on dentine. We washed for a double time (i.e., 30-60 seconds). The surface was dried without dehydrating dentine. The adhesive was then applied: Gluma Comfort Bond + Desensitizer with Venus and Prime&Bond NT with Esthet-X; each adhesive was applied in three layers with a Microbrush® then light-cured for 40 seconds with Visilux 2™(3M) curing lamp. We continued by stratifying composite increments of maximum 2 mm in height, each light-cured for 20 seconds. Finishing touches were executed with diamond fine-grit bur (Komet®) on a high-speed handpiece and Sof-Lex Pop-on (3M) disks.

-*In vitro* study

The *in vitro* experiment began with the preparation of 14 disk-shaped specimens (6mm in diameter and 2mm in height) of the two composites used in our restorations: 7 were made up with Venus, (Heraeus-Kulzer®) and 7 with Esthet-X (Dentsply®). The specimens were obtained from a precision impression of an absolutely smooth surface of a stainless steel block. The impression material Coltoflax™ (Coltène) was used to obtain the disk specimens in a sterilized cap. After polymerization the specimens were hydrated in sterile Phosphate Saline Buffer (PBS) for 30 minutes. Meanwhile a broth (Jordon’s basal medium) for *S. mutans* as prepared, made up from two solutions mixed after individual autoclave cycles. Solution A contained: 5g/l of trypticase peptone, 5g/l of yeast extract, 5g/l of K2HPO4, 0.05g/l of Na2CO3 in 0.05ml of saline Jordan solution. To prepare 10 ml of Jordan’s saline solution 1.15g of MgSO4 x 7H2O; 0.75g of MnSO4 x 4H2O; 0.068g of FeSO4 x 7H2O, diluted in 10 ml of H2O are necessary. Solution B of Jordan medium is made of saccharose 2%. After separate autoclave cycles of 20 minutes at 121°C, solution A and B are mixed to obtain the broth.

1 ml aliquots of Jordan’s basal medium were dispensed into 24 wells of a sterile plate (Greiner labortechnik®) for 24h. The 14 disk-shaped specimens of composite were than placed in the same pits and incubated with a suspension of *S. mutans* NTCT 10449 of a known quantity (1ml, 6.6x108 CFU/ml, 2.2 McFarland) for 24h at 37°C. The broth and *S. mutans* suspension were put into 10 wells without composite disk specimens as controls. At the end of the incubation, the bacterial amount within the wells was estimated with a qualitative evaluation of the total *S. mutans* growth. In order to do that 10 µl of suspension were taken from each well and cultivated on agar-blood medium plates. After overnight incubation at 37°C, the number of colonies was counted. The remained suspensions were taken and evaluated with a turbidimeter.

The specimens were washed with 1 ml of PBS and bacteria adherent to their surfaces were removed with trypsin. The content of every well were collected and analysed with the same turbidimeter at a 590nm wavelength.

## Results

The results obtained from plaque samples by bacterial culture showed that all patients had kept their normal oral microbiological state. None of the patients showed growth of *S. mutans* neither before or after restoration, a week and a month later, with no differences between the two composites and the control group.

PCR was negative for *S. mutans* in all samples. Figure 1 shows some of the PCR results: the only positive sample is the positive *S. mutans* control.

**Figure 1:** Agarose gel electrophoresis of some samples of the study group: all samples were negative: on the left the “M” lane represents the marker,“K+” the positive control of *S. mutans*.

The *in vitro* results are summarized in  Table 1 and  Table 2.

**Table 1:** Optical density of broths picked up from the wells after incubation of 24h.

**Table 2:** Turbidimetric results of trypsin collected bacteria: no differences in adhesion between the two composites.

 Table 1 shows the turbidimetric evaluations in McFarland of suspensions picked up from the pits after 24h incubation.

In all wells for both composites (Venus and Esthet-X) no differences were elicited about the growth of *S.mutans*, while in the controls wells, which contained only broth and *S. mutans* suspension, the turbidimeter detected a greater growth of *S. mutans*. The initial optical density of the broth was of 2,2 MF (1 McFarland corresponds to 3x108 CFU/ml). Non parametric Mann-Whitney U-test was used as statistical analysis. The results of group 1 (Esthet-X) were compared with group 2 (Venus) and no statistical differences were found (*p*>0.06), while the gap was significant (*p*<0.05) between groups 1 and 3 (controls); the same results were obtained between groups 2 and 3.

 Table 2 shows the turbidimetric evaluation of trypsin collected bacteria to verify the adhesion of *S. mutans* to disk-shaped composite specimens. The initial turbidimeter value was 0.49MF. The same non parametric statistical test was used to analyse the differences of *S. mutans* adhesion: no significant gaps were found, (*p*>0.05).

## Discussion

Abfractions, non-carious cervical lesions determined by bite overloading on teeth, are lesions which can be found frequently by dentists and patients are more worried about both aesthetics and symptomatology.

Composite resins are nowadays the most used restoration materials in dentistry because of their simple employment, versatility, mechanical and physical properties and extremely optical time-serving. Although a material capable of substituting the lost dental tissues is not available yet, last generation composites are absolutely the best presidium in restorative dentistry, even for abfractions.

In this study we zeroed in on the effects of composite materials towards bacterial plaque and particularly on *S. mutans*, in non-carious cervical lesions. The amount of dental plaque adhering on artificial restorative materials could actually cause secondary decay, ending up into a failure of the restorative therapy.

The results obtained revealed that restorations with composite materials do not modify the state of bacterial microflora of the non carious cervical lesions observed. The traditional bacterial culture analysis in different mediums (Mitis salivarius, Mitis salivarius with bacitracin and Blood-Agar) in both anaerobiosis and aerobiosis, of plaque samples (collected from the perimeters of cervical lesions, before and after their restoration) showed no significant qualitative or quantitative microbiological differences. Comparing cultured plates of consecutive samples of a same patient, actually, there were no different species of bacteria and no increase in growth of determined species. Even comparing plates from patients of the study group with plates from patients of the control group (free from cervical lesions or carious lesions), no differences were found. The most frequent bacteria species were *S. salivarius*, *S. sanguis* and Gram positive bacteria, belonging to a normal bacterial microflora.

The presence of *S. salivarius* and of notorious competitors of S. mutans could explain the reason why in none of the patients *S. mutans* was found. The abfractions included in our study were non-carious lesions, so we were quite sure not to find *S. mutans*, main aetiopathogenetic decay factor, in the first plaque sample. This finding was confirmed by mean of both traditional microbiological culture and PCR. Polymerase Chain Reaction is a very sensible and specific test, able to detect, the presence or absence of a target bacteria, viable or not viable, even in a small sample of plaque. The results obtained by PCR corroborated the data of traditional bacterial culture, revealing the absence of *S. mutans*, both before and after abfraction restoration by both composites. We did not found *S. mutans* even a week and a month later. Similar conclusions were found in other previous studies, although with different experimental models (14,15).

Our results are related to a multifactorial pathology (such as decay), so these data could depend not only on a good quality of restoration or on the material used themselves, but on the characteristics of the host too, as oral hygiene, low carbohydrates diet, buffer quality of the saliva and actual absence of *S. mutans*.

In the *in vitro* experiment, we focused on the effects of composite material towards growth of *S. mutans* and its adhesion to the material composite, without considering superficial roughness. The plates cultured with the broths picked up from the wells in which the disk-shaped specimens of composite were conserved did not give significant differences if compared with the controls. Turbidmeter evaluation did not show statistically relevant differences between the two composites tested, but it elicited a significant difference between the broths with the specimens and the broths without composite specimens. Turbidimetric results of the cultured broths and of trypsinized *S. mutans*, using a non- parametric statistic test (Mann Whitney U-test), pointed out a significant difference between the two experimental groups compared with control group respectively (*p*<0.05).

No differences were found between the two composites groups (*p*>0.06). Additionally, *S. mutans* adhesion to the two resins was not different (*p*>0.05); these data are similar to the results (0.5%-2%) obtained in a previous experience, in which different materials were used, by Poggio *et al.* (16) 2003.

In this study a relevant consideration was elicited: composite materials, *in vivo*, do not modify plaque composition of non carious cervical lesions to a potential cariogenic plaque. Furthermore *in vitro* they seem to slow down the growth or even to be bacteriostatic versus *S. mutans* and versus plaque microflora. It might probably depend *in vivo* on good host conditions: self-cleansing of abfraction sites (buccal surfaces) or low carbohydrate diet, good oral hygiene and good finishing and fitting of restoration. *In vitro*, the reduction in the growth of *S. mutans* could be due to the chemical nature of composite resins it self.
